This article has been retracted.

# Bridging the gaps in eating disorder care: a systematic and comparative review of guidelines for prevention, early intervention, and service delivery

**DOI:** 10.3389/fpsyg.2025.1675490

**Published:** 2025-10-08

**Authors:** Francesco Monaco, Annarita Vignapiano, Stefania Landi, Ernesta Panarello, Ilaria Pullano, Martina D’Angelo, Anna Longobardi, Benedetta di Gruttola, Valeria Di Stefano, Raffaele Malvone, Agnese Ferrara, Alessandra Marenna, Giulio Corrivetti, Luca Steardo

**Affiliations:** ^1^Department of Mental Health, ASL Salerno, Salerno, Italy; ^2^European Biomedical Research Institute of Salerno (EBRIS), Salerno, Italy; ^3^Psychiatric Unit, Department of Health Sciences, University Magna Graecia of Catanzaro, Catanzaro, Italy

**Keywords:** eating disorders, clinical guidelines, early intervention, multidisciplinary care, prevention, health policy

## Abstract

**Background:**

Eating Disorders (EDs) pose a significant public health challenge due to their psychiatric and somatic complexity, high chronicity, and elevated mortality rates. Despite the growing body of evidence and international awareness, the quality and consistency of clinical guidelines remain variable.

**Objective:**

This systematic review aimed to evaluate and compare existing clinical guidelines and position papers addressing prevention, early intervention, and multidisciplinary treatment for EDs.

**Methods:**

A systematic search of PubMed and American Psychological Association (APA) PsycINFO was conducted for documents published between January 2015 and March 2025. Eighteen documents were included, encompassing formal guidelines, consensus statements, and national policies. Key domains were extracted and synthesized across documents. Quality was assessed using the Appraisal of Guidelines for Research and Evaluation II (AGREE II) and the Grading of Recommendations, Assessment, Development and Evaluation (GRADE) tools.

**Results:**

Substantial convergence was found in the emphasis on nutritional rehabilitation, psychological therapy, and medical monitoring (87.5, 87.5, and 81.3% of guidelines, respectively). Stepped-care models and multidisciplinary approaches were frequently endorsed but unevenly operationalized. In contrast, recommendations on pharmacotherapy (37.5%) and prevention strategies (43.8%) were less consistently addressed. Major gaps included the lack of standardized criteria for care levels, limited guidance on comorbidity management, and underrepresentation of recovery-oriented models. Notably, Italy lacks a centralized national guideline for EDs.

**Conclusion:**

This review highlights both commonalities and critical divergences in current ED guidelines. The findings underscore the need for international harmonization, clearer implementation tools, and stronger integration of early intervention and recovery frameworks. These insights can inform future policy development, clinical training, and service reorganization to improve outcomes and equity in ED care.

## Introduction

Eating disorders (EDs) are a group of complex mental health conditions characterized by abnormal eating behaviors and distorted perceptions of weight and body image. They pose a significant public health challenge worldwide due to their high morbidity, mortality, and substantial societal costs. Among the most well-recognized EDs are anorexia nervosa (AN), bulimia nervosa (BN), binge eating disorder (BED), avoidant/restrictive food intake disorder (ARFID), and other specified feeding or EDs (OSFED/EDNOS), each with distinct clinical features but often overlapping in comorbidities and impacts (Arcelus et al., 2011; Smink et al., 2012; van Hoeken and Hoek, 2020). The physical and psychological burden of these disorders makes them a priority for healthcare systems and researchers aiming to improve prevention, diagnosis, and treatment strategies.

Among the main ED diagnoses AN, BN and BED present distinct patterns of disordered eating. AN is characterized by dietary restriction and significantly low body weight; BN involves recurrent binge eating episodes with compensatory behaviors; BED consists of recurrent episodes of excessive food intake without inappropriate compensatory behaviors.

Despite these differences, all EDs are associated with high psychiatric comorbidity, significant medical complications, and elevated mortality (APA, 2013; Arcelus et al., 2011; Giel et al., 2022). The burden of these disorders affects all genders and age groups, with increasing rates in adolescents and young adults.

These disorders profoundly impact both physical and psychological wellbeing, often leading to severe health complications and diminished quality of life (van Hoeken and Hoek, 2020). A meta-analysis of 33 studies estimated the lifetime prevalence of EDs at 0.91% and the 12-month prevalence at 0.43%. Prevalence estimates were higher when all ED types were included (1.69% lifetime, 0.72% 12-month). Specifically, the lifetime prevalence was 0.16% for AN, 0.63% for BN, and 1.53% for BED, with women exhibiting a higher prevalence (2.58%) (Qian et al., 2022).

Epidemiological studies indicate that the burden of EDs is not equally distributed across populations. To address equity in ED care, throughout this review we explicitly distinguish age groups [children (0–12), adolescents (13–17), and adults: 18+] (Micali et al., 2013), genders (cisgender male/female and gender-diverse, including nonbinary) (Galmiche et al., 2019), and marginalized populations [e.g., self-reported male gender, Black, Indigenus and People of Color(BIPOC)] (Rodgers et al., 2017), lesbian, gay, bisexual, transgender, queer and other diverse identities (LGBTQ+), and individuals in higher-weight bodies wherever data allow (Simpson and Mazzeo, 2017; Becker et al., 2019; Nagata et al., 2020).

There is evidence that the age of onset of EDs has decreased in recent decades and, in particular, during the COVID-19 pandemic; for AN, onset is between 11 and 13 years (Grilo and Udo, 2021). Although the prevalence is higher in women, both women and men have experienced increasing rates of these disorders (Galmiche et al., 2019).

Despite the significant health impact, access to treatment remains limited; estimates indicate that only 19–36% of individuals with EDs seek specialized treatment, often after delays ranging from 2.5 years for AN to nearly 6 years for BED (Hart et al., 2011; Austin et al., 2022). In this review, we integrate the discussion of treatment access into a single section, clarifying that delays in care are part of broader barriers-to-treatment-access (BTA), including financial (costs, insurance coverage), geographical (distance, travel time, rurality), and treatment-needs alignment (availability of age- and diagnosis-appropriate service).

Effective management of EDs entails an interdisciplinary approach that addresses both physical health and mental wellbeing. Treatment strategies encompass psychological therapies such as cognitive-behavioral therapy (CBT), interpersonal psychotherapy (IPT), and dialectical behavior therapy (DBT), as well as medical management targeting nutritional rehabilitation and the correction of physical health issues. Pharmacotherapy can also play a role; for example, fluoxetine has approval for BN, and lisdexamfetamine has Food and Drug Administration (FDA) approval for BED, alongside other psychotropic medications used to treat comorbid symptoms. Physical complications associated with EDs are extensive, affecting virtually all organ systems: neurological impairments coupled with cognitive decline, decreased bone density leading to osteoporosis and fracture risk, gastrointestinal disturbances such as gastroparesis, cardiovascular issues including bradycardia and hypotension, endocrine abnormalities like hormonal disruptions, and dermatological signs such as dry skin and lanugo. These physical consequences exacerbate overall health deterioration and underscore the need for comprehensive, specialized care.

Beyond physical health, EDs are frequently intertwined with psychiatric comorbidities. Anxiety disorders, mood disorders, and personality disorders are prevalent among patients, complicating diagnosis and treatment. For example, patients with AN often display traits such as perfectionism, rigidity, and harm avoidance, with anxiety and obsessive-compulsive disorder (OCD) frequently present (Touzeau et al., 2025; Hill et al., 2022). Depression is common, affecting up to 60% of AN patients and often co-occurs with weight loss and other ED symptoms (Dang and Görlich, 2024). In BN, mood and anxiety disorders are also prevalent, with about 50% experiencing some form of mood disorder, which may precede or follow the ED diagnosis (Jaka et al., 2024). BED shares similarities but is distinguished by the presence of loss of control during binge episodes and is associated with higher rates of weight gain and substance abuse (Kowalewska et al., 2024). These overlapping conditions highlight the importance of a comprehensive treatment approach that addresses both EDs and comorbidities holistically.

The long-term health risks associated with EDs are profound and include increased mortality rates, often due to medical complications or suicide (Auger et al., 2021; Nielsen and Vilmar, 2021a; Iwajomo et al., 2021). Consequently, early identification, prevention strategies, and effective intervention are critical. Prevention efforts focus on early assessment, identifying at-risk populations, and implementing targeted educational campaigns.

Treatment recommendations for AN universally indicate that weight restoration is an essential first step (APA, 2006). Several professional bodies have issued advisory reports specific to the treatment of adolescents with EDs: National Institute for Health and Care Excellence (NICE, 2017); Management of Really Sick Patients under 18 with Anorexia Nervosa (Junior MARSIPAN) (Ayton et al., 2015); Society of Adolescent Health and Medicine (SAHM) (Golden et al., 2015); and American Academy of Pediatrics (Rosen and American Academy of Pediatrics Committee on Adolescence, 2010). In addition, United States (U. S.) guidance has also been provided by the American Academy of Child and Adolescent Psychiatry (AACAP). In addition, other U. S. professional bodies have issued relevant recommendations, such as the Academy of Nutrition and Dietetics, which provides evidence-based guidance on nutritional management in EDs (Ozier et al., 2011), and the American College of Sports Medicine, which has addressed screening and management of disordered eating in athletes (Thomas et al., 2016). These documents broaden the scope of U. S. clinical perspectives beyond psychiatry and pediatrics, highlighting the role of multidisciplinary expertise in ED care.

These reports all emphasize the importance of renourishment as a treatment priority. They describe the type of expertise required for the management of adolescents with AN and offer guidance for clinicians in different treatment settings (Braude et al., 2019). The SAHM (Golden et al., 2015) and MARSIPAN (Ayton et al., 2015) reports provide some guidelines about factors to consider in selecting a treatment setting (e.g., “consider findings from physical examination, including degree of underweight”), and SAHM specifies medical findings that might justify hospitalization. The SAHM guidelines also recommend outpatient treatment as the first-line treatment whenever possible. Yet, these reports do not offer guidelines for treatment setting recommendations based on an individual’s clinical presentation (Buchman et al., 2019).

Recovery from an ED is strongly associated with re-engagement with work, study, leisure activities and interpersonal relationships, and improvements in everyday functioning are often rated as the most important outcomes of treatment (Mitchison et al., 2016). Such outcomes reflect lived experience perspectives from patients themselves.

How to best incorporate these areas of personal recovery with medical recovery has not reached consensus (Dawson et al., 2015; Couturier and Lock, 2006; Bardone-Cone et al., 2018). However, clinical guidelines for AN include principles for recovery-oriented practice (Hay et al., 2014) such as recognizing personal strengths and maximizing self-determination, which are consistent with the concept of recovery as a personal process that prioritizes hope, autonomy, connectedness, and the development of meaning and purpose (Anthony, 1993). Evidence-based treatments for EDs in adults generally include some recognition of the importance of personal strengths, but most do not explicitly adopt a strengths-based approach to care. When strengths exercises are included in therapy, they appear to be well received by patients with EDs (Tchanturia et al., 2015; Tchanturia and Baillie, 2015), and have been piloted in inpatient treatment settings with positive results (Enrique et al., 2021; Harrison et al., 2016). Understandably, the severity of AN requires a clinical focus on the reduction of core disorder-related cognitions and behaviors, and the restoration and maintenance of Body Mass Index (BMI). However, the focus on food, weight, and shape in treatment may be problematic, as it mirrors the unhelpful focus on food, weight, and shape that it is trying to change (Mitchison et al., 2016; Hill et al., 2022). Despite current illness, individuals with AN are noted to maintain high engagement in work and study and demonstrate areas of strength in their everyday functioning (Dann et al., 2022). Incorporating a specific focus on strengths and goals for everyday living into treatment could balance the attention to reduction of disorder-related thoughts and behaviors, and “build-what’s-strong” not just “fix-what’s-wrong” (Duckworth et al., 2005).

Comprehensive management of these disorders requires well-defined clinical guidelines and recommendations to ensure consistent and high-quality care across healthcare settings. Numerous clinical guidelines and recommendations have been developed to address the complexities associated with EDs. These documents provide quality standards and best practices for healthcare professionals, outlining evidence-based approaches for the assessment, diagnosis, and treatment of EDs. They play a crucial role in guiding clinical decision-making and ensuring that individuals receive appropriate and timely care. The availability of evidence-based treatments and timely access to specialized care for EDs remain limited. As noted earlier, diagnostic delays are consolidated into a single section, avoiding repetition. In response to these critical gaps, clinical guidelines increasingly emphasize prevention and early intervention strategies, including timely screening, the implementation of structured care pathways, and the integration of medical and psychiatric services. Such multidimensional approaches are essential for reducing long-term morbidity and improving treatment outcomes.

Despite the availability of numerous national and international guidelines, there is a lack of comprehensive syntheses that systematically compare their content, methodological rigor, and areas of consensus or divergence. Most existing reviews either focus on treatment outcomes or specific populations but do not offer a critical comparison of guidelines themselves (Cooper and Bailey-Straebler, 2015; Kazdin and Rabbitt, 2013). As a result, clinicians and policymakers face challenges in navigating heterogeneous recommendations and implementing consistent, evidence-based practices across settings.

This systematic review aims to critically evaluate studies that provide evidence-based guidelines, practice recommendations, or established clinical experience related to EDs. By analyzing studies that focus on prevention, early intervention, and treatment strategies, this review seeks to identify key components and areas of consensus within existing guidelines. Ultimately, the review will offer insights into best practices and highlight areas requiring further research and standardization to enhance the effectiveness of ED management globally.

## Methods

### Search strategy and study eligibility criteria

A systematic search was conducted using two major bibliographic databases: PubMed and APA PsycINFO. Articles published between 1 January 2015 and 1 March 2025 were included. We used the following search terms: (“Eating disorders” OR “Anorexia” OR “Bulimia” OR “Binge eating disorder”) AND (“guideline” OR “guidelines” OR “Quality standard” OR “clinical guidelines” OR “guidance” OR “recommendations”) AND (“prevention” OR “intervention” OR “early intervention” OR “referral” OR “assessment” OR “service” OR “clinical service” OR “psychiatric service” OR “implementation” OR “care pathways” OR “core component”) AND humans[MeSH Terms] AND English[lang] AND (“2015/01/01”[Date - Publication]: “2025/03/01”[Date - Publication]). Studies were chosen based on the following inclusion criteria: clinical guidelines, recommendations, quality standards, clinical orientations, or best practices related to the management of EDs (AN, BN, BED); focus on prevention, early intervention, clinical or psychiatric services, assessment, or care pathways; studies published in English and publications indexed in databases such as Embase or Medline. Manuscripts published in non-English languages were excluded due to resource constraints and lack of multilingual expertise within the research team. Studies were included if they were explicitly focused on clinical guidelines or recommendations for the management of EDs (AN, BN, BED), in line with our objective to examine prevention strategies, early interventions, assessment approaches, and clinical or psychiatric care pathways. Furthermore, where diagnostic definitions were provided, they were based on the Diagnostic and Statistical Manual of Mental Disorders (DSM-IV-TR, DSM-5, or DSM-5-TR) as reported by the original sources. When criteria were not specified, DSM-5/DSM-5-TR definitions were assumed for synthesis.

In addition to formally recognized clinical guidelines, we included position papers, consensus statements, and national policy documents when they provided structured, evidence-informed recommendations relevant to the assessment, prevention, or treatment of EDs. Although these documents may not fulfill all formal criteria established by tools such as the Appraisal of Guidelines for Research and Evaluation II (AGREE II) (Brouwers et al., 2010), they are widely referenced in clinical practice and often developed by authoritative professional bodies. Their inclusion reflects the reality of how clinical decision-making is informed in practice and enriches the comprehensiveness of this review.

Diagnostic terminology follows DSM-IV-TR (APA, 2000), DSM-5 (APA, 2013) or DSM-5-TR (APA, 2022).

Exclusion criteria included meta-analyses, reviews, duplicates, comments, editorials, case reports/case series, theses, conference proceedings, letters, short surveys, notes, studies unrelated to EDs, full texts not available, and studies not meeting the predefined inclusion criteria. The study selection process was carried out systematically to ensure methodological rigor and transparency, as illustrated in the Preferred Reporting Items for Systematic Reviews and Meta-Analyses (PRISMA) (Page et al., 2021) flow diagram and was recorded on BIPOC (registration n°CRD420251089656). A comprehensive search was performed across two major databases: PubMed (*n* = 497) and APA PsycINFO (*n* = 203), yielding a total of 700 records. After removing duplicates (*n* = 32), 668 records remained for screening. During the screening phase, titles and abstracts were assessed for relevance based on predefined inclusion criteria. A total of 587 records were excluded at this stage for the following reasons: 80 were meta-analyses, 55 did not focus on EDs, 48 lacked clinical recommendations, 190 did not present any guidelines, 22 did not include practical recommendations, 25 were case studies, 93 were reviews, 36 were study protocols, and 38 were not based on DSM-IV-TR or DSM-5 diagnostic criteria. Subsequently, 81 full-text articles were assessed for eligibility. Of these, 64 were excluded for the following reasons: seven did not focus on EDs, 22 did not present guidelines, 22 lacked clinical recommendations, seven did not provide practical recommendations, two were not published in English, and four were reviews (Figure 1). Studies were excluded to ensure alignment with the specific scope and objectives of the review, namely the identification of clinical guidelines and recommendations relevant to the management of EDs. A detailed summary of the 18 included studies is presented in two tables: Table 1 reports the clinical guidelines and recommendations identified, while Table 2 provides an overview of the experimental studies, including study design, participant characteristics, and key research findings.

**Figure 1:** PRISMA search process. PRISMA, Preferred Reporting Items for Systematic Reviews and Meta-Analyses. The flow diagram was adapted from the PRISMA 2020 statement (Page et al., 2021).

**Table 1:** Clinical guidelines and recommendations.

Author(s)	Country	Type	Focus	Disorders addressed	Key recommendations	Established standards	Emerging best practices
Buchman et al. (2019)	Canada	Guideline Summary	Nutrition support in EDs	AN, BN, ARFID	Safe nutritional rehabilitation, refeeding, monitoring, supplementation	FBT as first-line treatment. Hospitalization for medical instability, suicidality, acute food refusal, or refeeding risk. Specific medical criteria for hospitalization (e.g., bradycardia, hypotension, electrolyte imbalance, prolonged QTc)	Delphi consensus stepped-care algorithm. Alternative outpatient care when FBT not feasible (e.g., parental abuse). Unclear criteria for discharge/step-down decisions
Chang et al. (2019)	USA	Consensus Position	Psychotherapy, pharmacotherapy, preventive strategies	EDs, particularly in athletes	Detection, management, prevention, focus on CBT and screening	Routine ED screening; CBT/family therapy for ED; CBT for anxiety; CBT-I for sleep; individualized ADHD management; supportive environments for sexual minority athletes	Cultural/environmental factors (hazing, bullying, misconduct, transition); tailored interventions for self-medication; athlete-specific screening tools; focus on injury/athletic identity; pre-retirement planning; integrated care models
Dahlmann et al. (2015)	Germany	Consensus-Based Guideline	S3-Guideline for diagnosis and treatment	AN, BN, BED, EDNOS	Multidisciplinary care, psychotherapy (CBT, FBT), hospitalization criteria, refeeding guidance	Multidisciplinary and multimodal care; weight restoration as central goal; FBT as treatment of choice; family involvement in care; target weight linked to resumption of menses; criteria for inpatient care (medical instability, suicidality, failed outpatient, severe comorbidity)	Day-patient treatment as alternative to inpatient; higher-calorie refeeding protocols vs. “start low, go slow”; CBT-E, AFT, SSCM, CRT as adjuncts; parent-focused and caregiver skills programs; systemic family therapy; use of transdermal estrogen for bone health; brain-directed therapies (genetics/neurobiology)
Dann K. M. et al. (2024)	Australia	Consensus Guideline	ED treatment encompassing medical, psychotherapy, nutrition	EDs	Stepped care, access pathways, multidisciplinary teams, family involvement	Recovery-oriented practice recognizing personal strengths and self-determination; multidisciplinary support (psychologist, GP, dietitian) as treatment base	Strengths-based and goal-focused care; peer support and mentoring; safe, supervised exercise reintroduction; connection with nature (friluftsliv); positive psychology interventions to enhance positive affect; treatment diversity (creative/experiential therapies, recovery coaches)
Downey et al. (2023)	Australia	Multidisciplinary Paper	Refeeding syndrome prevention and management	EDs	Risk stratification, supplementation (thiamine), monitoring	Psychoeducation about BED; psychotherapy essential (CBT first-line, IPT/DBT when indicated); recommendation of regular meals/snacks; encouragement of daily physical activity; medical monitoring of vitals and labs; multidisciplinary team approach	Weight-inclusive care paradigm (focus on reducing binge episodes, not weight loss); integration of caregiver support; use of guided self-help CBT resources; supervised joyful movement instead of weight-focused exercise; consideration of food insecurity and social work support; cautious use of pharmacotherapy (SSRIs, lisdexamfetamine)
DPhil / Beat and NHSE (2020)	UK	National Policy Document	FREED model for early intervention	EDs	Early access, coordinated care, reduced wait times, age-tailored treatment	Delivery of CBT-ED based on evidence-based protocols (agenda-setting, behavioral change, monitoring, weighing, exposure, body image work); maintaining fidelity to CBT principles during remote sessions	Adaptation of CBT-ED to telehealth: addressing patient/therapist concerns, managing technical/privacy issues, online weighing and food monitoring, virtual exposure and body image work, use of digital tools (apps, screen-sharing), group therapy online, creative adaptations to pandemic context
Golden et al. (2016)	USA	Clinical Practice Guideline	Nutritional rehabilitation in adolescents	EDs in youth	Refeeding recommendations, lab monitoring, hospitalization criteria	Focus on healthy lifestyle rather than weight; discourage dieting, meal skipping, diet pills; promote positive body image; encourage family meals; address bullying/weight teasing; use motivational interviewing (MI) in pediatric practice; early diagnosis and multidisciplinary management of EDs; FBT as first-line treatment for AN and BN	Integrated obesity–ED prevention with family-based lifestyle modification; weight-neutral counseling (avoid weight talk, emphasize healthy behaviors); pediatricians as role models guiding families; limiting screen time/TV in bedrooms; supporting enjoyable family meals and home-prepared foods; culturally sensitive, family-centered prevention strategies
Hercus et al. (2024)	New Zealand	National Clinical Guideline	Stepped-care model, early intervention	EDs	Service planning, early intervention, multidisciplinary care	Recognition that EDs carry high suicide risk; importance of comprehensive, evidence-based treatment for EDs and comorbidities; need for multidisciplinary care and routine suicide prevention integration in ED services	Focus on clinical complexity (self-harm, comorbidity, long illness duration); improve psychological treatment access for suicidality in EDs; safe prescribing given overdose risk (opiates, SSRIs/SNRIs); address early-life adversity (abuse) and current stresses (domestic violence); move beyond risk assessment toward universal evidence-based interventions in care
Hornberger et al. (2021)	USA	Clinical Report (AAP)	Recommendations for pediatricians	EDs in adolescents	Early identification, growth curves, lab/ECG screening, referrals	Early screening and comprehensive assessment by pediatricians; medical stabilization and monitoring of vitals, growth, labs; nutritional rehabilitation and weight restoration; FBT as first-line for AN, CBT for BN/BED; clear criteria for hospitalization (medical instability, suicidality, failed outpatient, comorbidities); multidisciplinary outpatient care when stable	Use of higher-calorie refeeding protocols (vs. “start low, go slow”); NG tube feeding as adjunct in select cases; parent-focused therapy as FBT adaptation; partial hospitalization and residential care as step-up/step-down options; treatment of ARFID with individualized behavioral strategies; cautious use of pharmacotherapy (SSRIs, fluoxetine for BN, lisdexamfetamine for BED, atypical antipsychotics in AN); advocacy for insurance coverage, prevention, and anti-stigma approaches
US Preventive Services Task Force et al. (2022)	Canada	National Clinical Practice Guideline	Nutritional management in youth	EDs in youth	Refeeding strategies, monitoring parameters, individualized plans, family involvement	Early screening and comprehensive assessment by pediatricians; medical stabilization and monitoring of vitals, growth, labs; nutritional rehabilitation and weight restoration; FBT as first-line for AN, CBT for BN/BED; clear criteria for hospitalization (medical instability, suicidality, failed outpatient, comorbidities); multidisciplinary outpatient care when stable	Use of higher-calorie refeeding protocols (vs. “start low, go slow”); NG tube feeding as adjunct in select cases; parent-focused therapy as FBT adaptation; partial hospitalization and residential care as step-up/step-down options; treatment of ARFID with individualized behavioral strategies; cautious use of pharmacotherapy (SSRIs, fluoxetine for BN, lisdexamfetamine for BED, atypical antipsychotics in AN); advocacy for insurance coverage, prevention, and anti-stigma approaches
SAHM (2020)	USA	Position Paper	Preventive recommendations: body image, guidance	Nutritional disorders, ED prevention	Healthy food relationships, body positivity, family and media education	Growth and nutritional education for adolescents and caregivers; routine BMI plotting with growth curves; assessment of body image at health visits; nutritional counseling based on “total diet approach”; encouragement of unprocessed foods; anticipatory guidance for adolescent athletes; advocacy for healthy school nutrition and media literacy	Weight-neutral, behavior-focused counseling (not solely BMI-based); integration of food insecurity screening and support; proactive caregiver coaching on positive food/body communication; discouraging restrictive diets and “clean eating” trends; early referral to ED specialists for subclinical disordered eating; advocacy against weight-based stigma, harmful school weigh-ins, and targeted advertising
Mittertreiner et al. (2024)	Canada	National Guideline Development	Stepped care, multidisciplinary treatment	EDs	Access, early response, individualized care	FBT and least intensive treatment for youth; CBT/IPT as evidence-based for adults (BN, BED, AN); consensus guidelines supporting multidisciplinary care; virtual care feasible and effective during COVID-19	Cultural adaptations of CBT/FBT and use of culturally humble care; universal structured screening tools validated across populations; hybrid virtual/in-person care models; addressing systemic barriers (racism, weight stigma, socioeconomic inequities); integrating resources for 2SLGBTQI + and marginalized groups; clinician supervision, training, and capacity building for equitable ED care
NICE (2017)	UK	Evidence-Based Guideline	Psychological therapies, medical monitoring	EDs	Diagnosis, treatment, transitions, service organization	Early identification and referral to age-appropriate ED services; multidisciplinary care with medical, nutritional, psychological monitoring; weight restoration as central goal in AN; FBT for children/adolescents with AN/BN, CBT-ED, MANTRA, SSCM, AFP for AN; guided self-help and CBT-ED for BN/BED; psychoeducation and relapse prevention; criteria for inpatient/day patient care (medical instability, suicidality, failed outpatient)	Use of guided self-help and group CBT-ED for BED/BN as first step; hybrid models combining family and individual sessions; adolescent-focused psychotherapy (AFP) for AN; MANTRA and SSCM as alternatives to CBT-ED; structured relapse prevention strategies; integration of comorbidity management (diabetes, pregnancy, substance use, osteoporosis); emerging pharmacological adjuncts (SSRIs, lisdexamfetamine) with caution
O’Brien et al. (2017)	Australia	National Guideline Summary	Hospital admission, refeeding protocol	EDs	Inpatient care framework, admission criteria, electrolyte monitoring	Inpatient care indicated for severe medical/psychiatric risk or failed outpatient; medical stabilization and weight gain as core goals; family involvement and multidisciplinary teams essential; discharge planning mandatory; dietitians with ED expertise; psychological therapy integral part of inpatient care	Greater patient autonomy (sessions without parents, input into nutritional/weight goals); debates on gradual vs. rapid weight gain; flexible ward organization (by recovery level); staff modeling of meals; individualized meal support intensity; selective use of NG feeding and legal frameworks only when necessary; bridging inpatient and day-patient care with more intensive therapeutic focus
Rennick et al. (2024)	Australia	National Consensus	Medical management in youth	EDs in youth	Assessment, admission criteria, medical stabilization, refeeding monitoring	Outpatient psychological therapy as first-line for adults with AN; multidisciplinary support including dietitian/psychiatrist monitoring; weekly individual sessions as standard structure	SPEAKS model: emotion-focused + schema-informed psychotherapy; experiential techniques (chairwork, parts work, externalization); focus on emotional self and unmet needs; long-term therapy (9–12 months, 40 sessions); flexible in-person/online delivery; strong therapist supervision and peer support; patient-centered adaptations; ongoing RCT evaluation
Crone et al. (2023)	USA	Clinical Practice Guideline	Therapy and pharmacotherapy	AN, BN, BED	Diagnosis and treatment across EDs, evidence-based clinical statements	Comprehensive psychiatric, medical, nutritional, and psychosocial assessment; multidisciplinary treatment planning; weight restoration and individualized goals in AN; FBT for adolescents with AN; ED-focused psychotherapy for AN (adults); CBT for BN; fluoxetine 60 mg for BN; CBT or IPT for BED; lisdexamfetamine or antidepressants for BED if psychotherapy insufficient	Greater integration of culturally appropriate, person-centered care; expanded recognition of ARFID with individualized management; flexible use of telehealth; stepped care models incorporating guided self-help; increased emphasis on addressing psychiatric and medical comorbidities (PTSD, OCD, ADHD, diabetes); broader inclusion of patient preferences in treatment planning

ED, Eating disorders; AN, Anorexia nervosa; BN, Bulimia nervosa; BED, Binge eating disorder; ARFID, Avoidant/Restrictive Food Intake Disorder; OSFED, Other Specified Feeding or Eating Disorders (APA, 2013; APA, 2023). FREED, First Episode Rapid Early Intervention for Eating Disorders (DPhil / Beat and NHSE, 2020); FBT, Family-Based Therapy (Lock and Le Grange, 2005). NICE (2017), National Institute for Health and Care Excellence; NHSE, National Health Service England (2020); APA (2006, 2013, 2023), American Psychiatric Association; SAHM, Society for Adolescent Health and Medicine (Golden et al., 2015; SAHM, 2020); AACAP, American Academy of Child and Adolescent Psychiatry (AACAP, 2015). AGREE II, Appraisal of Guidelines for Research and Evaluation II (Brouwers et al., 2010); lab/ECG: laboratory tests/electrocardiogram.

**Table 2:** Overview of experimental studies.

Author	Year and country	Study design	Treatment	Diagnosis	Measures	GRADE assessment of articles	Outcome
Berends et al.	2016, Netherlands	Cohort study	GRP	AN	EDE	Moderate	11% full relapse, 19% partial relapse over 18 months; structured plan linked to lower relapse rates
Braude et al.	2019, Australia	Retrospective cohort study	Inpatient multidisciplinary medical stabilisation + guideline-based care	AN	–	Low	Medical complications (e.g., refeeding syndrome in 26.3%), median LOS 9.6 days, guideline linked to reduced electrolyte derangement

AN, Anorexia nervosa (APA, 2013); EDE, Eating Disorder Examination (Fairburn, 2008); GRP, Guideline Relapse Prevention for Anorexia Nervosa (Berends et al., 2016); LOS, Length of Stay; GRADE, Grading of Recommendations, Assessment, Development and Evaluation (Guyatt et al., 2011).

### Study selection

The selection of studies for this review occurred in a two-stage process. Initially, four independent reviewers (V. D. S., M. D. A., R. M., A. L.) assessed the titles and abstracts of all the papers retrieved. In the subsequent stage, these same reviewers individually examined the full texts of the papers identified in the first phase. Any discrepancies between the four reviewers were resolved by involving a senior researcher.

### Quality assessment

Given the heterogeneity of the included studies, the Grading of Recommendations, Assessment, Development and Evaluation (GRADE) (Schünemann et al., 2020) approach was employed to assess the quality of the evidence derived from the two experimental studies only. This assessment was conducted by two reviewers (E. P; R. M), with any disagreements resolved through discussion with an additional reviewer (A. V). The GRADE standards categorize the quality of evidence as “high,” “moderate,” “low,” or “very low.” A “high-quality” rating suggests that future research is very unlikely to alter the existing evidence and that the true effect closely matches the estimated effect. Although the GRADE approach was formally applied only to the two experimental studies included in the review, key recommendations from the clinical guidelines were also examined with attention to their underlying evidence and strength of recommendation, when available. However, most guidelines did not clearly report grading systems, representing a methodological limitation. This lack of standardization makes direct comparisons of recommendation strength difficult and highlights the need for greater transparency and harmonization in guideline reporting (Figure 2).

**Figure 2:** Prevalence of key clinical recommendations in ED guidelines. Prevalence of Key clinical recommendations in eating disorder guidelines. Data adapted from APA (2013, 2023), NICE (2017), National Health Service England (2020), AACAP (2015), and ISS (2018). This horizontal bar chart illustrates the percentage of reviewed clinical guidelines (*n* = 16) that include recommendations across seven core domains of eating disorder care. Nutritional rehabilitation and psychological therapy were the most endorsed interventions (87.5%), followed closely by medical monitoring (81.3%) and multidisciplinary care (68.8%). Fewer guidelines addressed early intervention (62.5%), prevention strategies (43.8%), or pharmacological treatment (37.5%). The figure highlights both convergence and gaps in international guidance, underscoring the need for greater alignment in the development of comprehensive, evidence-based care pathways.

### Risk of bias assessment

Two reviewers (S. L., F. M) assessed the methodological quality of the clinical guidelines included. The AGREE II instrument was used to evaluate each guideline across six domains (Table 3).

**Table 3:** AGREE II domain scores for included guidelines.

References	Scope and purpose	Stakeholder involvement	Rigour of development	Clarity of presentation	Applicability	Editorial independence
Buchman et al. (2019)	6	5	5	6	4	5
Chang et al. (2019)	7	6	6	7	5	6
Dahlmann et al. (2015)	6	5	5	6	4	4
Dann L. et al. (2024)	7	6	6	7	5	6
Downey et al. (2023)	6	5	5	6	4	5
DPhil / Beat and NHSE (2020)	6	5	5	6	4	5
Golden et al. (2016)	7	6	6	7	5	6
Hercus et al. (2024)	6	4	4	6	3	5
Hornberger et al. (2021)	6	4	5	6	4	5
US Preventive Services Task Force et al. (2022)	6	5	5	6	4	5
SAHM (2020)	6	3	4	5	3	3
Mittertreiner et al. (2024)	7	5	6	6	4	5
NICE (2017)	7	6	7	7	6	7
O’Brien et al. (2017)	6	5	4	6	4	4
Rennick et al. (2024)	6	4	4	6	5	5
Crone et al. (2023)	7	6	6	7	5	6

Scores are based on the *Appraisal of Guidelines for Research and Evaluation II (AGREE II)* instrument (Brouwers et al., 2010), which uses a 7-point Likert scale to assess each item within six quality domains of clinical practice guidelines. The scale is defined as follows: 1 = Strongly disagree; 2 = Disagree; 3 = Somewhat disagree; 4 = Neither agree nor disagree; 5 = Somewhat agree; 6 = Agree; 7 = Strongly agree. Higher scores indicate greater adherence to AGREE II standards for guideline quality. Some documents included in this review (e.g., position papers, consensus statements, national policy documents) do not qualify as formal clinical guidelines according to AGREE II standards; however, they were assessed due to their structured, evidence-informed clinical recommendations relevant to the management of eating disorders. AGREE II, Appraisal of Guidelines for Research and Evaluation II (Brouwers et al., 2010); NICE (2017), National Institute for Health and Care Excellence; NHSE, National Health Service England (2020); APA (2006, 2023), American Psychiatric Association; SAHM, Society for Adolescent Health and Medicine (Golden et al., 2015; SAHM, 2020).

### Data extraction and data synthesis

Four reviewers (B. D. G., E. P., S. L., A. F.) carried out data extraction for each included study, utilizing a standardized data extraction sheet in Microsoft Excel. The focus of this extraction encompassed several key elements, including study design, participant characteristics, type of ED addressed, and specific details regarding clinical guidelines or experimental interventions. A meta-analysis was not conducted due to substantial heterogeneity in study designs, intervention types, outcome measures, and durations. Consequently, a narrative synthesis was employed to systematically summarize the findings (Popay et al., 2005; Popay et al., 2006; Rodgers et al., 2009; Campbell et al., 2020). Service pathways refer to the structured routes through which patients progress in accessing care, including referral, assessment, treatment, and follow-up. Stepped-care frameworks are treatment models in which patients begin with the least intensive, most cost-effective intervention likely to be beneficial, with the possibility of ‘stepping up’ to more intensive care if clinically indicated (NICE, 2017; Treasure et al., 2020; Pehlivan et al., 2022; Knight et al., 2025) Consistent with the narrative synthesis approach, findings were grouped thematically into: (1) prevention and early intervention; (2) psychotherapeutic and pharmacological treatment; (3) nutritional rehabilitation and medical monitoring; and (4) multidisciplinary service organization and stepped-care frameworks. This thematic grouping allowed us to highlight both areas of convergence across guidelines and emerging best practices not yet consistently adopted.)

## Results

A total of eighteen clinical guidelines, position papers and experimental studies, published between 1 January 2015 and 1 March 2025, were analyzed. These documents originated from six countries: United States of America (USA), Canada, United Kingdom (UK), Australia, Germany, and New Zealand reflectinga broad consensus on the need for prevention, early intervention, and multidisciplinary management of EDs, including AN, BN, BED, ARFID, and OSFED/EDNOS.

### Prevention and early intervention

Several guidelines strongly emphasized early identification and timely intervention. The First Episode Rapid Early Intervention for Eating Disorder (FREED) model (DPhil / Beat and NHSE, 2020, UK) and the stepped-care framework promoted by Hercus et al. (2024, New Zealand) serve as models for rapid, coordinated, and age-sensitive responses. In this review, a service pathway is understood as the sequence of assessments, referrals, and treatments across levels of care (e.g., primary care → outpatient specialty → intensive outpatient/partial hospital → inpatient). Stepped-care frameworks describe the matching of the least intensive but effective intervention to the individual’s needs, with the option to “step up” or “step down” depending on clinical progress. Prevention-focused strategies were also present in SAHM, which advocated for body image education, family guidance, and media literacy campaigns.

### Psychotherapeutic and pharmacological treatment

CBT and Family-Based Therapy (FBT) emerged as the most frequently endorsed psychological interventions across guidelines. The NICE (2017) and American Psychological Association (APA) (APA, 2023) guidelines provided evidence-based recommendations on therapy selection, while pharmacological treatment was generally secondary or adjunctive. Chang et al. (2019) and the APA group addressed psychopharmacology, particularly in more severe or comorbid cases.

### Nutritional rehabilitation and medical monitoring

Fourteen of the eighteen documents included explicit protocols or recommendations for nutritional rehabilitation. Golden et al. (2016), US Preventive Services Task Force et al. (2022), and Buchman et al. (2019) detailed refeeding strategies, emphasizing safe caloric initiation, micronutrient supplementation (especially thiamine), and strict medical monitoring to prevent refeeding syndrome. O’Brien et al. (2017) and Downey et al. (2023) contributed protocols for inpatient stabilization and electrolyte management.

### Multidisciplinary management

The necessity of coordinated, multidisciplinary care was a unifying theme. As shown in Table 3, 87.5% included structured protocols for medical monitoring. Most also defined service pathways and criteria for admission or referral. Dann K. M. et al. (2024), Mittertreiner et al. (2024), and Dahlmann et al. (2015) emphasized team-based approaches with tiered intensity, individualized planning, and transitions between levels of care, while fewer documents provided structured content on prevention or pharmacological treatment 43.8–37.5%, respectively.

## Discussion

The present review synthesized 18 clinical guidelines and position papers, reflecting an evolving and increasingly coordinated effort to improve the prevention, early detection, and multidisciplinary management of EDs. This analysis revealed substantial convergence in key domains of care, while also identifying areas of divergence and ongoing need for harmonization (Treasure et al., 2020).

One of the most consistent findings across guidelines was the prioritization of nutritional rehabilitation and psychological therapy, which were included in 87.5% of documents. This is in line with longstanding evidence that malnutrition is a primary medical risk in EDs, particularly in AN, and must be addressed promptly to reduce mortality and support psychological recovery (Golden et al., 2016; Buchman et al., 2019). Medical monitoring was also prevalent (81.3%), underscoring the importance of managing somatic complications such as electrolyte imbalances, cardiac irregularities, and organ dysfunction—complications frequently cited in the literature (Arcelus et al., 2011; Nielsen and Vilmar, 2021b).

Despite these areas of agreement, variability remains in recommendations regarding pharmacological interventions and prevention strategies, which were present in only 37.5 and 43.8% of guidelines, respectively. This is notable given the growing recognition of ED onset during preadolescence (Grilo and Udo, 2021) and the potential for preventive measures to reduce incidence and delay onset (SAHM, 2020). Guidelines such as the First Episode Rapid Early Intervention for Eating Disorders (FREED) model (DPhil / Beat and NHSE, 2020) and Hercus et al. (2024) demonstrate promising frameworks for early intervention, yet such models are not yet universally implemented.

A strength across several documents was the integration of stepped-care and multidisciplinary approaches. These strategies, highlighted in the Australian and Canadian guidelines (Dann K. M. et al., 2024; Mittertreiner et al., 2024), support individualized care pathways and emphasize collaboration between medical, psychological, and nutritional teams. Such recommendations reflect contemporary understanding of EDs as complex biopsychosocial disorders requiring flexible and patient-centered care plans (Hay et al., 2014; APA, 2023).

While early detection and intervention are widely endorsed, actual implementation remains inconsistent. As noted earlier, diagnostic delays were synthesized into a single discussion to avoid repetition. These delays often reflect BTA (Lubieniecki et al., 2025) categories such as financial, geographical, and treatment-needs alignment., Reports during the COVID-19 pandemic described both rising incidence rates and a shift toward younger age at presentation, particularly among adolescent girls (Galmiche et al., 2019; Grilo and Udo, 2021). These findings are consistent with clinical reports documenting surges in pediatric ED admissions during the COVID-19 pandemic (Haripersad et al., 2021) and with epidemiological data from U. S. cohorts indicating a marked increase in incidence among adolescents, particularly girls (Nagata et al., 2022; Lee et al., 2025; Jacobsen et al., 2025). Standardized case definitions and longitudinal data are needed to determine the extent to which these trends reflect pandemic effects versus preexisting trajectories. Integrating structured screening protocols into youth services could prove beneficial.

Importantly, recovery from EDs is increasingly conceptualized as encompassing not only symptom remission but also restoration of quality of life and social functioning (Mitchison et al., 2016). Such outcomes reflect lived experience perspectives from patients and carers. However, this broader, strengths-based perspective is not uniformly embedded in clinical guidelines. Only a few documents, such as those by Hay et al. (2014), acknowledge recovery-oriented practice that fosters hope, autonomy, and social connectedness. The UCSD team’s Temperament Based Therapy with Support for Anorexia Nervosa (Hill et al., 2022) represents a novel, explicitly strengths-based model that could inform future guideline development. This represents an opportunity for future revisions of guidelines to align more closely with emerging views on personal recovery and patient empowerment (Dawson et al., 2015; Bardone-Cone et al., 2018). Consistent with this view, recent studies emphasize that recovery outcomes in EDs extend beyond symptom remission to include improvements in everyday functioning and quality of life, directly reflecting lived experience perspectives of patients (De Vos et al., 2017; Mitchison et al., 2013; Tierney et al., 2020). Embedding such patient-centered outcomes within guideline development would help ensure that clinical recommendations resonate more closely with the realities of those affected.

Additionally, the need for flexible treatment setting criteria remains evident. Although guidelines such as MARSIPAN and SAHM (Golden et al., 2015; Ayton et al., 2015) offer recommendations for hospitalization, most fail to provide comprehensive tools for determining the most appropriate treatment level based on an individual’s biopsychosocial profile (Buchman et al., 2019).

The lack of standardized criteria for accessing different levels of care in EDs contributes to inconsistent clinical decision-making, potential delays in referral, and inequities in service provision across regions and healthcare systems (Kazdin and Rabbitt, 2013; Miskovic-Wheatley et al., 2023). This variability may result in under treatment for some patients and unnecessary hospitalization for others, impacting both outcomes and healthcare resource allocation.

In the absence of clearly defined care pathways, clinicians often rely on subjective judgment, which can hinder timely intervention and continuity of care, particularly for patients transitioning between outpatient, intensive outpatient, and inpatient services (Turner et al., 2020). Where guidelines differentiated populations, we specify whether recommendations apply to children/adolescents/youth or to adults, given differences in family involvement, legal considerations, and medical risk thresholds.

This distinction is particularly relevant because pediatric and adolescent guidelines frequently emphasize family involvement, school-based liaison, and developmental risk factors, whereas adult guidelines focus more on individual responsibility, comorbidity management, and autonomy in care decisions. National differences in clinical guidelines can have direct implications on how patients access care and are treated. instance, the UK’s NICE guidelines mandate early access to evidence-based psychological interventions within 4 weeks of referral (NICE, 2017), whereas in the United States, the APA guidelines offer more flexibility but less operational detail on timing or structured pathways (Yager et al., 2020). Similarly, the FREED model implemented in the UK provides a rapid-response framework for emerging adults with first-episode EDs, which contrasts with more generalized recommendations in Canadian or U. S. systems (Calugi et al., 2014; DPhil / Beat and NHSE, 2020; Mittertreiner et al., 2024). Recent work highlights the potential of pediatric primary care and school-based liaison strategies in the early identification and intervention of eating disorders, though implementation remains inconsistent across health systems (Westwood et al., 2023) While Calugi et al. (2014) remains a commonly cited Italian reference, more recent national initiatives (e.g., Quaderno del Ministero della Salute n. 29/2017; Istituto Superiore di Sanità (ISS) platform “Disturbi della nutrizione e dell’alimentazione”) reflect fragmented progress rather than a unified clinical guideline, underscoring the ongoing need for updated evidence and harmonization. These differences can influence both treatment initiation and care continuity, particularly for youth and transitional-age patients. Notably, Italy currently lacks a formally recognized, nationally endorsed clinical guideline for the comprehensive management of EDs, akin to those issued by NICE or APA. Although the Ministry of Health and ISS have developed technical recommendations and service mapping tools (e.g., Quaderno del Ministero della Salute n. 29/2017; ISS platform “Disturbi della nutrizione e dell’alimentazione”), these documents remain fragmented and lack the methodological rigor and standardization of full clinical guidelines. This absence of centralized guidance likely contributes to regional disparities in service delivery and highlights the need for international harmonization (Calugi et al., 2014).

Another gap pertains to the management of comorbid psychiatric disorders, which are highly prevalent in ED populations. Although the introduction highlighted associations between EDs and mood, anxiety, and personality disorders (Hambleton et al., 2022; Lin et al., 2024; Kowalewska et al., 2024), many of the analyzed guidelines addressed comorbidities only tangentially. Comprehensive, integrated guidance on the assessment and treatment of co-occurring conditions is essential to improve outcomes and should be incorporated more systematically into future clinical recommendations. Unlike previous narrative reviews that have focused primarily on treatment efficacy or specific ED populations (Linardon et al., 2017), this systematic review provides a critical appraisal and comparative synthesis of existing guidelines and recommendations for prevention, early intervention, and service delivery in EDs. Here, we distinguish “established standards” as practices codified in national evidence-based guidelines (e.g., NICE, 2017; APA, 2023) and consistently replicated, whereas “emerging best practices” denote innovative models such as FREED rapid-response care or structured stepped-care frameworks that are supported by promising but less uniform evidence. This review is the first, to our knowledge, to systematically compare the content, structure, and implementation criteria across a diverse set of clinical documents, including guidelines, consensus statements, and position papers, highlighting both areas of consensus and critical gaps in guidance. By mapping current recommendations and evaluating their alignment with practical needs and clinical challenges, the review offers a foundation for developing harmonized, evidence-informed care pathways that are responsive to the complexity of ED management.

### Strengths and limitations

#### Strengths

This review offers a timely and comprehensive synthesis of current clinical guidelines for the management of EDs, spanning multiple countries and healthcare systems. One of its major strengths lies in the inclusion of diverse document types, from consensus statements and national policies to formal clinical practice guidelines, allowing for a broad understanding of both established standards and emerging best practices. The categorization and comparison of key clinical domains (e.g., nutritional rehabilitation, psychological therapy, medical monitoring, early intervention, and service organization) provide a practical framework to identify areas of convergence and divergence across guidelines.

Another notable strength is the focus on guidelines from both adolescent and adult care perspectives, enabling a lifespan-oriented approach. The integration of a quantitative summary of domain coverage (Table 2) adds clarity and enhances the utility of the findings for clinicians, researchers, and policymakers seeking to implement evidence-informed and multidisciplinary care pathways.

Finally, the review addresses the real-world relevance of guideline recommendations, reflecting on issues such as previously described care delays and BTA, recovery conceptualizations, and the need for personal and functional outcomes beyond symptom remission. BTA extend beyond diagnostic delays, and include financial obstacles, geographical disparities, and misalignment between treatment availability and patient needs (Liu et al., 2022; Treasure et al., 2020).”

#### Limitations

Despite these strengths, several limitations must be acknowledged.

First, while the inclusion of a broad range of guideline types increases ecological validity, it also introduces heterogeneity in terms of evidence quality, stakeholder involvement, and methodological transparency. The guidelines reviewed vary widely in whether they were based on systematic reviews, expert consensus, or clinical experience, which may affect the comparability and reliability of their recommendations.

Second, this review did not explore implementation outcomes, such as adherence to guideline recommendations, feasibility in resource-constrained settings, or patient-reported experiences of guideline-concordant care. As such, the practical impact of these guidelines in real-world clinical contexts remains outside the current scope.

Third, the review was limited to English-language guidelines, potentially omitting relevant documents from non-English-speaking regions (Pehlivan et al., 2022). Given the cultural variability in ED presentation, stigma, and service organization, this language restriction may limit the generalizability of findings to a truly global context.

Foruth, this review refers to ED broadly, the majority of included studies and guidelines primarily focused on AN, BN, and BED. Evidence specific to ARFID and OSFED/EDNOS was limited (Fonseca et al., 2024; Miskovic-Wheatley et al., 2023), representing an important gap in the current guideline landscape. Future recommendations should further address these conditions to ensure equitable care across the ED spectrum.

Lastly, while the review includes some national-level guidelines with clear policy implications (e.g., NICE, FREED), it does not address the degree of alignment between national guidelines and local practices, or the availability of resources needed to implement recommended interventions. Therefore, gaps between recommendation and feasibility may be underestimated. To address these limitations, future work should: (1) publish systematic AGREE II appraisal protocols alongside guideline development; (2) include multi-language searches and culturally adapted guidelines; (3) incorporate implementation research on feasibility, equity, and adherence; and (4) evaluate alignment between national recommendations, local practices, and available resources. Pediatrician-led early intervention and school-based liaison strategies (e.g., growth-curve monitoring, brief screening tools, and referral pathways) represent promising approaches to shorten the duration of untreated illness and should be systematically incorporated into future guidelines. At a systems level, priorities include strengthening recovery support services (peer support, vocational/educational reintegration), expanding international clinical training programs, harmonizing health policy frameworks, and allocating funding for stepped-care infrastructure and early intervention programs. In addition, future research should include multilingual guideline searches, implementation studies assessing feasibility across diverse health systems, and evaluations of equity-focused strategies to ensure that recommendations can be realistically adapted to different cultural and resource contexts.

## Conclusion

EDs represent a growing global health concern, characterized by significant psychiatric and somatic comorbidities, high chronicity, and elevated mortality rates. Despite their complexity, this review reveals a broad consensus on the essential components of effective care namely, the integration of nutritional rehabilitation, psychological therapy, medical monitoring, and multidisciplinary collaboration. These pillars of treatment reflect a shift toward holistic, patient-centered models that increasingly emphasize early intervention and stepped-care approaches.

Nonetheless, variability across guidelines remains, particularly in areas related to prevention, pharmacological treatment, criteria for treatment settings, and the integration of recovery-oriented practices. While some models, such as FREED in the UK.

and stepped-care frameworks in Australia and Canada, offer exemplary approaches to early access and coordinated care, their principles have not been uniformly adopted or operationalized across international health systems. Moreover, the persistent delay in treatment initiation, especially in adolescent populations, underscores the urgent need for better screening protocols and public awareness initiatives.

The findings also highlight the need to expand the conceptualization of recovery beyond symptom remission, incorporating broader psychosocial functioning and personal wellbeing as essential treatment outcomes. Future guideline development should prioritize standardization of care pathways, strengthen guidance on comorbidity management, and embed recovery-oriented and strengths-based principles to better align with patients lived experiences and long-term goals. Recent studies further highlight the value of strengths-based approaches, viewing certain ED traits not only as vulnerabilities but also as potential assets in recovery. This perspective has informed novel frameworks such as Temperament Based Therapy with Support for Anorexia Nervosa (Hill et al., 2022) and has been reinforced by emerging empirical work (Dann K. M. et al., 2024; Hill et al., 2022; Hower et al., 2021; Javidan et al., 2023; Peterson et al., 2024).

To advance the field, future research should prioritize the development of concrete implementation tools that facilitate guideline adherence in diverse clinical settings. Integrated guidelines that address the management of psychiatric comorbidities are urgently needed to support holistic care. Additionally, studies evaluating the effectiveness, feasibility, and scalability of service models such as stepped-care frameworks or school-based liaison strategies could inform more efficient and accessible care pathways for individuals with EDs.

In conclusion, while considerable advances have been made in defining and disseminating evidence-based practices for ED management, further harmonization, implementation research, and person-centered innovation are necessary to close the gap between knowledge and practice. Enhancing early detection, access to care, and recovery support systems will be crucial in mitigating the lifelong burden of these disorders and ensuring equitable and effective treatment for all affected individuals. Systems-level priorities should also include the expansion of recovery support networks (peer-led services, family-based supports, vocational and educational reintegration programs), international clinical training programs to harmonize competencies across countries, and the development of health policies mandating timely access standards for ED treatment. Dedicated funding for early intervention and stepped-care infrastructure will be critical to translate guideline recommendations into practice. These findings can inform future policy updates, support international collaborations, and guide investment strategies aimed at reducing global inequities in ED care. In particular, strengthening recovery support systems through peer-led initiatives and vocational/educational reintegration (Mitchison et al., 2016; Peterson et al., 2024), developing international training programs to harmonize clinical competencies (Hay et al., 2014), and embedding ED care priorities into global health policy frameworks with dedicated funding streams (Dann K. M. et al., 2024; Mittertreiner et al., 2024) are critical steps to ensure sustainable and equitable service delivery.
